# Analysis of Pull-In Instability of Geometrically Nonlinear Microbeam Using Radial Basis Artificial Neural Network Based on Couple Stress Theory

This article has been retracted.

**DOI:** 10.1155/2014/571632

**Published:** 2014-04-17

**Authors:** Mohammad Heidari, Ali Heidari, Hadi Homaei

**Affiliations:** ^1^Mechanical Engineering Group, Islamic Azad University, Aligudarz Branch, P.O. Box 159, Aligudarz, Iran; ^2^Faculty of Engineering, Shahrekord University, P.O. Box 115, Shahrekord, Iran

## Abstract

The static pull-in instability of beam-type microelectromechanical systems (MEMS) is theoretically investigated. Two engineering cases including cantilever and double cantilever microbeam are considered. Considering the midplane stretching as the source of the nonlinearity in the beam behavior, a nonlinear size-dependent Euler-Bernoulli beam model is used based on a modified couple stress theory, capable of capturing the size effect. By selecting a range of geometric parameters such as beam lengths, width, thickness, gaps, and size effect, we identify the static pull-in instability voltage. A MAPLE package is employed to solve the nonlinear differential governing equations to obtain the static pull-in instability voltage of microbeams. Radial basis function artificial neural network with two functions has been used for modeling the static pull-in instability of microcantilever beam. The network has four inputs of length, width, gap, and the ratio of height to scale parameter of beam as the independent process variables, and the output is static pull-in voltage of microbeam. Numerical data, employed for training the network, and capabilities of the model have been verified in predicting the pull-in instability behavior. The output obtained from neural network model is compared with numerical results, and the amount of relative error has been calculated. Based on this verification error, it is shown that the radial basis function of neural network has the average error of 4.55% in predicting pull-in voltage of cantilever microbeam. Further analysis of pull-in instability of beam under different input conditions has been investigated and comparison results of modeling with numerical considerations shows a good agreement, which also proves the feasibility and effectiveness of the adopted approach. The results reveal significant influences of size effect and geometric parameters on the static pull-in instability voltage of MEMS.

## 1. Introduction

Microelectromechanical systems (MEMS) are widely being used in today's technology. So investigating the problems referring to MEMS owns a great importance. One of the significant fields of study is the stability analysis of the parametrically excited systems. Parametrically excited microelectromechanical devices are ever increasingly being used in radio, computer, and laser engineering [1]. Parametric excitation occurs in a wide range of mechanics, due to time-dependent excitations, especially periodic ones; some examples are columns made of nonlinear elastic material, beams with a harmonically variable length, parametrically excited pendulums, and so forth. Investigating stability analysis on parametrically excited MEM systems is of great importance. In 1995 Gasparini et al. [2] studied the transition between the stability and instability of a cantilevered beam exposed to a partially follower load. Applying voltage difference between an electrode and ground causes the electrode to deflect towards the ground. At a critical voltage, which is known as pull-in voltage, the electrode becomes unstable and pulls in onto the substrate. The pull-in behavior of MEMS actuators has been studied for over two decades without considering the casimir force [3–5]. Osterberg et al. [3, 4] investigated the pull-in parameters of the beam-type and circular MEMS actuators using the distributed parameter models. Sadeghian et al. [5] applied the generalized differential quadrature method to investigate the pull-in phenomena of microswitches. A comprehensive literature review on investigating MEMS actuators can be found in [6]. Further information about modeling pull-in instability of MEMS has been presented in [7, 8]. The classical continuum mechanics theories are not capable of prediction and explanation of the size-dependent behaviors which occur in micron- and sub-micron-scale structures. However, some nonclassical continuum theories such as higher-order gradient theories and the couple stress theory have been developed such that they are acceptably able to interpret the size dependencies. In 1960s some researchers such as Koiter [9], Mindlin and Tiersten [10], and Toupin [11] introduced the couple stress elasticity theory as a nonclassic theory capable of predicting the size effects with appearance of two higher-order material constants in the corresponding constitutive equations. In this theory, beside the classical stress components acting on elements of materials, the couple stress components, as higher-order stresses, are also available which tend to rotate the elements. Utilizing the couple stress theory, some researchers investigated the size effects in some problems [12]. Employing the equilibrium equation of moments of couples beside the classical equilibrium equations of forces and moments of forces, a modified couple stress theory was introduced by Yang et al. [13], with one higher-order material constant in the constitutive equations. Recently, size-dependent nonlinear Euler-Bernoulli and Timoshenko beams modeled on the basis of the modified couple stress theory have been developed by Xia et al. [14] and Asghari et al. [15], respectively. Rong et al. [16] present an analytical method for pull-in analysis of clamped-clamped multilayer beam. Their method is Rayleigh-Ritz method and assumes one deflection shape function. They derive the two governing equations by enforcing the pull-in conditions that the first and second order derivatives of the system energy functional are zero. In their model, the pull-in voltage and displacement are coupled in the two governing equations.

This paper investigates the pull-in instability of microbeams with a curved ground electrode under action of electric field force within the framework of von-Karman nonlinearity and the Euler-Bernoulli beam theory. The static pull-in voltage instability of clamped-clamped and cantilever microbeam is obtained by using MAPLE commercial software. The effects of geometric parameters such as beam lengths, width, thickness, gaps, and size effect are discussed in detail through a numerical study. The objective of this paper is to establish neural network model for estimation of the pull-in instability voltage of cantilever beams. More specifically, radial basis function (RBF) is used to construct the pull-in instability voltage. Effective parameters influencing pull-in voltage and their levels for training were selected through preliminary calculations carried out on instability pull-in voltage of microbeam. Networks trained by the same numerical data are then verified by some numerical calculations different from those used in training phase, and the best model was selected based on the criterion of having the least average values of verification errors. To the best of authors' knowledge, no previous studies which cover all these issues are available. To the authors' best knowledge, no previous studies which cover all these issues are available.

## 2. Preliminaries

In the modified couple stress theory, the strain energy density $\overset{-}{u}$ for a linear elastic isotropic material in infinitesimal deformation is written as [17]

(1) $$\begin{array}{c} \overset{-}{u}=\frac{1}{2}\left(\sigma_{ij}\varepsilon_{ij}+m_{ij}\chi_{ij}\right)\;\left(i,j=1,2,3\right), \end{array}$$

where

(2) $$\begin{array}{c} \sigma_{ij}=\lambda \varepsilon_{mm}\delta_{ij}+2\mu \varepsilon_{ij} \end{array}$$

(3) $$\begin{array}{c} \varepsilon_{ij}=\frac{1}{2}\left({\left(\nabla u\right)}_{ij}+{\left(\nabla u\right)}_{ij}^{T}\right) \end{array}$$

(4) $$\begin{array}{c} m_{ij}=2l^{2}\mu \chi_{ij} \end{array}$$

(5) $$\begin{array}{c} \chi_{ij}=\frac{1}{2}\left({\left(\nabla \theta \right)}_{ij}+{\left(\nabla \theta \right)}_{ij}^{T}\right), \end{array}$$

in which *σ*_*ij*_, *ε*_*ij*_, *m*_*ij*_, and *χ*_*ij*_ denote the components of the symmetric part of stress tensor *σ*, the strain tensor *ε*, the deviatoric part of the couple stress tensor *m*, and the symmetric part of the curvature tensor *χ*, respectively. Also, *u* and *θ* are the displacement vector and the rotation vector. The two Lame constants and the material length scale parameter are represented by *λ*, *μ*, and *l*, respectively. The Lame constants are written in terms of Young's modulus *E* and Poisson's ratio *ν* as *λ* = *νE*/(1 + *ν*)(1 − 2*ν*) and *μ* = *E*/2(1 + *ν*). The components of the infinitesimal rotation vector *θ*_*i*_ are related to the components of the displacement vector field *u*_*i*_ as [18]

(6) $$\begin{array}{c} \theta_{i}=\frac{1}{2}{\left(\mathrm{curl}\left(u\right)\right)}_{i}. \end{array}$$

For an Euler-Bernoulli beam, the displacement field can be expressed as

(7) $$\begin{array}{c} u_{x}=u\left(x,t\right)-z\frac{\partial w\left(x,t\right)}{\partial x},\;\;u_{y}=0,\\ \;\;u_{z}=w\left(x,t\right), \end{array}$$

where *u* is the axial displacement of the centroid of sections and *w* denotes the lateral deflection of the beam. The parameter ∂*w*/∂*x* stands for the angle of rotation (about the *y*-axis) of the beam cross-sections. Assuming the above displacement field, after deformation, the cross-sections remain plane and always perpendicular to the center line, without any change in their shapes. It is noted that parameter *z* represents the distance of a point on the section with respect to the axis parallel to *y*-direction passing through the centroid.

## 3. Governing Equation of Motion 

In this section, the governing equation and corresponding classical and nonclassical boundary conditions of a nonlinear microbeam modeled on the basis of the couple stress theory are derived. The coordinate system and loading of an Euler-Bernoulli beam have been depicted in Figure 1. In this figure, *F*(*x*, *t*) and *G*(*x*, *t*) refer to the intensity of the transverse distributed force and the axial body force, respectively, both as force per unit length.

By assuming small slopes in the beam after deformation, the axial strain, that is, the ratio of the elongation of a material line element initially in the axial direction to its initial length, can be approximately expressed by the von-Karman strain as

(8) εxx=∂u  x  ∂x+12(∂w∂x)2=∂u∂x−z∂2w∂x2+12(∂w∂x)2.

It is noted that finite deflection *w* is permissible and only it is needed that the slopes be very small. Hereafter, we use (8) for the axial strain, instead of the infinitesimal definition presented in (3). Substitution of (7) and (8) into (3)–(5) yields the nonzero components.

Also, combination of (6) and (7) gives [19]

(9) $$\begin{array}{c} \theta_{y}=-\frac{\partial w}{\partial x},\;\;\;\theta_{x}=\theta_{z}=0. \end{array}$$

Substitution of (9) into (5) yields the following expression for the only nonzero component of the symmetric curvature tensor:

(10) $$\begin{array}{c} \chi_{xy}=\chi_{yx}=-\frac{1}{2}\frac{\partial^{2}w}{\partial x^{2}}. \end{array}$$

It is assumed that the components of strains, rotations, and their gradients are sufficiently small. By neglecting Poisson's effect, substitution of (8) into (2) gives the following expressions for the main components of the symmetric part of the stress tensor in terms of the kinematic parameters:

(11) σxx=Eεxx=E(∂u∂x−z∂2w∂x2+12(∂w∂x)2),all  other  σij=0,

where *E* denotes the elastic modulus. In order to write the nonzero components of the deviatoric part of the couple stress tensor in terms of the kinematic parameters, one can substitute (10) into (4) to get

(12) $$\begin{array}{c} m_{xy}=-\mu l^{2}\frac{\partial^{2}w}{\partial x^{2}}, \end{array}$$

where *μ* and *l* are shear modulus and the material length scale parameter, respectively. To obtain the governing equations, the kinetic energy of the beam *T*, the beam strain energy due to bending and the change of the stretch with respect to the initial configuration *U*_*bs*_, the increase in the stored energy with respect to the initial configuration due to the existence of initially axial load *U*_*is*_, and finally the total potential energy *U* = *U*_*bs*_ + *U*_*is*_ are considered as follows:

(13a) $$\begin{array}{c} T=\frac{1}{2}\overset{L}{\underset{0}{\int }}\overset{}{\underset{A}{\int }}\rho \left\{{\left(\frac{\partial u}{\partial t}-z\frac{\partial^{2}w}{\partial t\partial x}\right)}^{2}+{\left(\frac{\partial w}{\partial t}\right)}^{2}\right\}dA\;dx \end{array}$$

(13b) U=12∫0L{EI(∂2w∂x2)2+EA(∂u∂x+12(∂w∂x)2)2     +N0[2∂u∂x+(∂w∂x)2]+μAl22(∂2w∂x2)}dx,

where *N*_0_, *I*, and *ρ* are the axial load, area moment of inertia of section about *y*-axis, and the mass density, respectively. The work done by the external loads acting on the beam is also expressed as

(13c) δW=∫0LF(x,t)δwdx+∫0LG(x,t)  δudx+(N^δu)|x=0x=L +(V^δw)|x=0x=L+(M^δ(∂w∂x))|x=0x=L +(P^hδ(∂u∂x+12(∂w∂x)2))|x=0x=L +(Q^hδ(∂2w∂x2))|x=0x=L,

where $\hat{N}$ and $\hat{V}$ represent the resultant axial and transverse forces in a section caused by the classical stress components acting on the section. The resultant axial and transverse forces are work conjugate to *u* and *w*, respectively. Also, ${\hat{P}}^{h}$ and ${\hat{Q}}^{h}$ are the higher-order resultants in a section, caused by higher-order stresses acting on the section. These two higher-order resultants are work conjugate to *ε*_*xx*_ = ∂*u*/∂*x* + 1/2(∂*w*/∂*x*)^2^ and ∂^2^ *w*/∂*x* ^2^, respectively. The parameter $\hat{M}$ is the resultant moment in a section caused by the classical and higher-order stress components. Now, the Hamilton principle can be applied to determine the governing equation:

(14) $$\begin{array}{c} \overset{t_{2}}{\underset{t_{1}}{\int }}\left(\delta T-\delta U+\delta W\right)dt=0, \end{array}$$

where *δ* denotes the variation symbol. By applying (13a), (13b), (13c), and (14), the governing equilibrium microbeam is derived as

(15) $$\begin{array}{c} S\frac{\partial^{4}w}{\partial x^{4}}-N\frac{\partial^{2}w}{\partial x^{2}}+\rho A\frac{\partial^{2}w}{\partial t^{2}}=F\left(x,t\right), \end{array}$$

where

(16) $$\begin{array}{c} N=N_{0}+\frac{EA}{2L}\overset{L}{\underset{0}{\int }}{\left(\frac{\partial w}{\partial x}\right)}^{2}dx\\ S=EI+\mu Al^{2}. \end{array}$$

If, in (15), *N* = 0, then the model of beam is called the linear equation (linear model) without the effect of geometric nonlinearity. The cross-sectional area and length of beam are *A* and *L*, respectively. *F*(*x*, *t*) is the electrostatic force per unit length of the beam. The electrostatic force enhanced with first order fringing correction can be presented in the following equation [20]:

(17) $$\begin{array}{c} F_{\text{elec}}\left(x,t\right)=\frac{\varepsilon_{0}BV^{2}}{2{\left(g-w\right)}^{2}}\left[1+0.65\frac{\left(g-w\right)}{B}\right], \end{array}$$

where *ε*_0_ = 8.854 × 10^−12^ C^2^ N^−1^ m^−2^ is the permittivity of vacuum, *V* is the applied voltage, *g* is the initial gap between the movable and the ground electrode, and *B* is width of beam. For clamped-clamped beam, the boundary conditions at the ends are

(18) $$\begin{array}{c} w\left(0\right)=0,\;\;\frac{dw\left(0\right)}{dx}=0;\\ w\left(L\right)=0,\;\;\frac{dw\left(L\right)}{dx}=0. \end{array}$$

For cantilever beam, the boundary conditions at the ends are

(19) $$\begin{array}{c} w\left(0\right)=0,\;\;\frac{dw\left(0\right)}{dx}=0;\\ \frac{d^{2}w\left(L\right)}{dx^{2}}=0,\;\;\frac{d^{3}w\left(L\right)}{dx^{3}}=0. \end{array}$$

Table 1 shows the geometrical parameters and material properties of microbeam.

In the static case, we have ∂/∂*τ* = 0 and ∂/∂*x* = *d*/*dx*. Hence, (15) is reduced to

(20) (EI+μAl2)d4wdx4−[N0+EA2L∫0L(dwdx)2dx]d2wdx2  =ε0BV22(g−w)2[1+0.65(g−w)B].

A uniform microbeam has a rectangular cross-section with height *h* and width *B*, subjected to a given electrostatic force per unit length. Let us consider the following dimensionless parameters:

(21) $$\begin{array}{c} \alpha =\frac{AL^{2}}{2I},\;\;\beta =\frac{\varepsilon_{0}BV^{2}L^{4}}{2g^{3}EI},\;\;\gamma =0.65\frac{g}{B},\;\\ \delta =\frac{\mu Al^{2}}{EI},\;\;\tilde{w}=\frac{w}{g},\;\;\tilde{x}=\frac{x}{L},\;\;\Gamma =\;\frac{N_{0}L^{2}}{EI}. \end{array}$$

In the above equations, the nondimensional parameter, *δ*, is defined as the size effect parameter. Also, *β* is nondimensional voltage parameter. The normalized nonlinear governing equation of motion of the beam can be written as [21]

(22) (1+δ)d4w~dx~−{Γ+α∫01(dw~dx~)2dx~}d2w~dx~2  =β(1−w~)2+γβ(1−w~).

## 4. Overview of Neural Networks

A neural network is a massive parallel system comprised of highly interconnected, interacting processing elements or nodes. Neural networks process through the interactions of a large number of simple processing elements or nodes, also known as neurons. Knowledge is not stored within individual processing elements, rather represented by the strengths of the connections between elements. Each piece of knowledge is a pattern of activity spread among many processing elements, and each processing element can be involved in the partial representation of many pieces of information. In recent years, neural networks have become a very useful tool in the modeling of complicated systems because they have an excellent ability to learn and to generalize (interpolate) the complicated relationships between input and output variables [22]. Also, the ANNs behave as model-free estimators; that is, they can capture and model complex input-output relations without the help of a mathematical model [23]. In other words, training neural networks, for example, eliminates the need for explicit mathematical modeling or similar system analysis.

### 4.1. Artificial Neural Network Models of Static Pull-In Instability of Beam

In this research radial basis function (RBF) neural network has been used for modeling the pull-in instability voltage of microcantilever beams. The radial basis network has some additional advantages such as rapid learning and low error. In particular, most RBFNs involve fixed basis functions with linearly unknown parameters in the output layer. In practice, the number of parameters in RBFN starts becoming unmanageably large only when the number of input features increases beyond 10 or 20, which is not the case in our study. Hence, the use of RBFN was practically possible in this research. In this paper, MATLAB Neural Network Toolbox (NNET) was used as a platform to create the networks [24].

#### 4.1.1. Radial Basis Function (RBF) Neural Network

The construction of a radial basis function (RBF) neural network in its most basic form involves three entirely different layers. A typical RBFN with *N* input and *M* output is shown in Figure 2. The input layer is made up of source nodes (sensory units). The second layer is a single hidden layer of high enough dimension, which serves a different purpose in a feedforward network. The output layer supplies the response of the network to the activation patterns applied to the input layer. The input units are fully connected though unit-weighed links to the hidden neurons, and the hidden neurons are fully connected by weighed links to the output neurons. Each hidden neuron receives input vector **X** and compares it with the position of the center of Gaussian activation function with regard to distance. Finally, the output of the *j*th-hidden neuron can be written as

(23) $$\begin{array}{c} A_{j}=\exp\left(-\frac{{||X_{i}-C_{j}||}^{2}}{S^{2}}\right), \end{array}$$

where **X**_*i*_ is an *N*-dimensional input vector, *C*_*j*_ is the vector representing the position of the center of the *j*th hidden neuron in the input space, and *S* is the standard deviation or spread factor of Gaussian activation function. The structure of a radial basis neuron in the hidden layer can be seen in Figure 3. Output neurons have linear activation functions and form a weighted linear combination of the outputs from the hidden layer:

(24) $$\begin{array}{c} Y_{k}=\overset{H}{\underset{j=1}{\sum }}w_{kj}A_{j}, \end{array}$$

where *Y*_*k*_ is the output of neuron *k*, *H* is the number of hidden neurons, and *w*_*kj*_ is the weight value from the *j*th hidden neuron to the *k*th output neuron. Basically, the RBFN has the properties of rapid learning, easy convergence, and low error, generally possessing the following characteristics.

1. It may require more neurons than the standard feedforward BP networks.
2. It can be designed in a fraction of the time that it takes to train the BP network.
3. It has excellent capability of representing nonlinear functions.

RBFN is being used for an increasing number of applications, proportioning a very helpful modeling tool [25].

## 5. Results and Discussion 

### 5.1. Static Pull-In Instability Analysis

When the applied voltage between the two electrodes increases beyond a critical value, the electric field force cannot be balanced by the elastic restoring force of the movable electrode and the system collapses onto the ground electrode. The voltage and deflection at this state are known as the pull-in voltage and pull-in deflection, which are of utmost importance in the design of MEMS devices. The pull-in voltage of cantilever and fixed-fixed beams is an important variable for analysis and design of microswitches and other microdevices. Typically, the pull-in voltage is a function of geometry variable such as length, width, and thickness of the beam and the gap between the beam and ground plane. To study the instability of the nanoactuator, (22) is solved numerically and simulated. To highlight the differences between linear and nonlinear geometry model results of Euler-Bernoulli microbeam, we first compare the pull-in voltage for fixed-fixed and cantilever beams with a length of 100 *μ*m, a width of 50 *μ*m, a thickness of 1 *μ*m, and two gap lengths. For a small gap length of 0.5 *μ*m (shown in Figure 4), we observe that linear and nonlinear geometry model give identical results. However, for a large gap length of 2 *μ*m (shown in Figure 5), we observe that pull-in voltage for fixed-fixed beam is significantly different. As shown in Figure 6, the difference in the pull-in voltage is even larger when a gap length of 4.5 *μ*m is considered. In Figures 7, 8, and 9, pull-in voltages of fixed-free beams are shown. It is evident that pull-in voltage of fixed-fixed beam is larger than fixed-free beam. More extensive studies for the cantilever beam with lengths varying from 100 to 500 *μ*m and thicknesses varying from 1 to 4 *μ*m are shown in Figures 10 and 11. The gap lengths used vary from 5 to 30 *μ*m. For gaps smaller than 15 *μ*m and lengths larger than 350 *μ*m, we observe that the pull-in voltages obtained with linear and nonlinear geometry model are very close. However, for large gaps (such as the 15 *μ*m case) and for short beams (such as the 100 *μ*m case), we observe that the difference in the pull-in voltage obtained with linear and nonlinear geometry model is not negligible. In Figures 12 and 13, we investigate the fixed-fixed beam example with lengths varying from 100 to 500 *μ*m and thicknesses varying from 0.5 to 2 *μ*m. We observe that, for all cases, the pull-in voltages obtained with linear model are with significant error (larger than 5.5%) compared to the pull-in voltages obtained with nonlinear geometry model. When the gap increases, the error in pull-in voltage with linear model increases significantly. Furthermore, contrary to the case of cantilever beams, the thickness has a significant effect on the error in pull-in voltages. The thinner the beam, the larger the error. Another observation is that the length of the beam has little effect on the error in pull-in voltage. This observation is also different from the case of cantilever beams. From the results, it is clear the linear model is generally not valid for the fixed-fixed beams case, except when the gap is very small, such as the 0.5 *μ*m case as shown in Figure 4. Effect of the size effect on the pull-in voltage of fixed-fixed and fixed-free beam is illustrated in Figures 12 and 13, respectively. These figures represent that the size effect increases the pull-in voltage of the nanoactuators. Figures 14 and 15 shows the pull-in voltage versus size effect for fixed-fixed beam and cantilever beam respectively.

### 5.2. Modeling of Static Pull-In Instability of Microcantilever Beam Using Neural Networks

Modeling of pull-in instability of microbeam with RBF neural network is composed of two stages: training and testing of the networks with numerical data. The training data consisted of values for beam length (*L*), gap (*g*), width of beams (*b*) and (*h*/*l*), and the corresponding static pull-in instability voltage (*V*_PI_). A total of 120 such data sets were used, of which 110 were selected randomly and used for training purposes whilst the remaining 10 data sets were presented to the trained networks as new application data for verification (testing) purposes. Thus, the networks were evaluated using data that had not been used for training. Training/testing pattern vectors are formed, each formed with an input condition vector and the corresponding target vector. We map each term to a value between −1 and 1 using the following linear mapping formula:

(25) $$\begin{array}{c} N=\frac{\left(R-R_{\min}\right)*\left(N_{\max}-N_{\min}\right)}{\left(R_{\max}-R_{\min}\right)}+N_{\min}, \end{array}$$

where *N* is normalized value of the real variable; *N*_min⁡_ = −1 and *N*_max⁡_ = 1 are minimum and maximum values of normalization, respectively; *R* is real value of the variable; *R*_min⁡_ and *R*_max⁡_ are minimum and maximum values of the real variable, respectively. These normalized data were used as the inputs and output to train the ANN. In other words, the network has four inputs of beam length (*L*), gap (*g*), width of beams (*b*) and (*h*/*l*) ratio, and one output of static pull-in voltage (*V*_PI_).  Figure 16 shows the general network topology for modeling the process.

Table 2 shows 10 numerical data sets, which have been used for verifying or testing network capabilities in modeling the process.

Therefore, the general network structure is supposed to be 4-n-1, which implies 4 neurons in the input layer, n neurons in the hidden layer, and 1 neuron in the output layer. Then, by varying the number of hidden neurons, different network configurations are trained, and their performances are checked. For training problem, equal learning rate and momentum constant of *η* = *α* = 0.9 were used [26]. Also, error stopping criterion was set at *E* = 0.01, which means training epochs continued until the mean square error fell beneath this value.

#### 5.2.1. RBF Neural Network Model (RBFNN)

Spread factor (*S*) value of Gaussian activation functions in the hidden layer of RBFNN is the parameter that should be determined by trial and error when using MATLAB neural network toolbox for designing RBF networks. It has to be larger than the distance between adjacent input vectors, so as to get good generalization, but smaller than the distance across the whole input space. Therefore, in order to have a network model with good generalization capabilities, the spread factor should be selected between 0.5 and 5.34. For training the RBF network, at first, a guess is made for the value of spread factor in the obtained interval. Also, the number of radial basis neurons is originally set as 1. At each iteration, the input vector that results in lowering most network training errors is used to create a radial basis neuron. Then, the error of the new network is checked, and if it is low enough, the training stopped. Otherwise, the next neuron is added. This procedure is repeated until the error goal is achieved, or the maximum number of neurons is reached [27, 28]. In the present case, it was found by trial and error that 20 hidden neurons, with the spread factor of 3, can give a model, which has the best performance in the verification stage.  Table 3 shows the effect of the number of hidden neurons on the RBF network performance. It is clear that although adding more than 20 hidden neurons makes the mean square error (MSE) training smaller, this deteriorates network's generalization capabilities with increasing the average verification errors instead of decreasing them. Therefore, the optimum number of radial basis neurons is 20. The selected network has the average errors of 4.55% in response to the 10 input verification calculations (Table 2) for *V*_PI_ with newrbe function.  Table 4 lists output values predicted by the RBF neural model and calculated ones in verification (testing) phase. Two functions, namely, newrbe and newrb, have been used for creating RBF networks.

From Tables 2 and 3, it is concluded that RBFN model has the total average error of 4.55%.  Figure 17 compares the pull-in voltages evaluated by the modified couple stress theory with *h*/*l* = 4, *g* = 1.05 *μ*m, *b* = 50 *μ*m, and *h* = 2.94 *μ*m with the result of RBF neural network. The pull-in voltages of the microcantilever versus parameter *h*/*l* for *b*/*g* = 50 are depicted in Figure 18, with two RBF functions. The correlation coefficients (*R*) are 0.997 for RBF model in simulating *V*_PI_.

## 6. Conclusions

The primary contributions of the paper are summarized as follows.

1. The RBF neural network is capable of constructing model using only numerical data, describing the static pull-in instability behavior.
2. RBF neural network, which possesses the privileges of rapid learning, easy convergence, and low error, has good generalization power and is accurate for this particular case. This selection was done according to the results obtained in the verification phase.
3. For cantilever beams, length has a significant effect on the error in pull-in voltages, while for fixed-fixed beams, the length has little effect on the error. On the other hand, for fixed-fixed beams, thickness has significant effect on the error in pull-in voltage, while for cantilever beams it has little effect.
4. The static pull-in instability voltages of clamped-clamped and cantilever beam are compared. For both clamped-clamped and cantilever beams, the pull-in voltage in nonlinear geometry beam model is bigger than in linear model.
5. For both fixed-fixed and cantilever beams by increasing of gap length, the pull-in voltage is significantly increased.
6. For both fixed-fixed and cantilever beams by increasing of thickness of beams, the pull-in voltage is significantly increased.
7. For both fixed-fixed and cantilever beams by increasing of length of beams, the pull-in voltage is significantly decreased.
8. By using modified couple stress theory, it is found that the dimensionless pull-in voltage of MEMS increases linearly due to the size effect. This emphasizes the importance of size effect consideration in design and analysis of MEMS.
9. The results have demonstrated the applicability and adaptability of the RBNN for analysis of instability static pull-in voltage of cantilever beams; also the newrbe function is more accurate and faster than newrb function.
10. When the ratio of *h*/*l* increases, the pull-in voltage predicted by modified couple stress theory and ANN is constant approximately.

The conclusion above indicates that the geometry of beam has significant influences on the electrostatic characteristics of microbeams that can be designed to tailor for the desired performance in different MEMS applications.

## Figures and Tables

**Figure 1:** An Euler-Bernoulli, loading, and coordinate system.

**Figure 2:** Radial basis function neural network.

**Figure 3:** Radial basis neuron.

**Figure 4:** Comparison of linear and nonlinear geometry model results for a fixed-fixed beam with a gap of 0.5 *μ*m.

**Figure 5:** Comparison of linear and nonlinear geometry model results for a fixed-fixed beam with a gap of 2 *μ*m.

**Figure 6:** Comparison of linear and nonlinear geometry model results for a fixed-fixed beam with a gap of 4.5 *μ*m.

**Figure 7:** Comparison of linear and nonlinear geometry model results for a fixed-free beam with a gap of 0.5 *μ*m.

**Figure 8:** Comparison of linear and nonlinear geometry model results for a fixed-free beam with a gap of 2 *μ*m.

**Figure 9:** Comparison of linear and nonlinear geometry model results for a fixed-free beam with a gap of 4.5 *μ*m.

**Figure 10:** Gap versus pull-in voltage for cantilever beams with a thickness of 1 *μ*m. For length that equals 100 *μ*m, the difference in pull-in voltage between linear and nonlinear geometry model is significant when the gap is larger than 15 *μ*m. For a length larger than 350 *μ*m, the pull-in voltages obtained with linear and nonlinear geometry model are identical.

**Figure 11:** Gap versus pull-in voltage for cantilever beams with a thickness of 4 *μ*m. For length that equals 100 *μ*m, the difference in pull-in voltage between linear and nonlinear geometry model is significant when the gap is larger than 15 *μ*m. For a length larger than 350 *μ*m, the pull-in voltages obtained with linear and nonlinear geometry model are identical.

**Figure 12:** Gap versus pull-in voltage for fixed-fixed beams with a thickness of 0.5 *μ*m. Observe the large difference in pull-in voltage obtained from linear and nonlinear geometry model of beam.

**Figure 13:** Gap versus pull-in voltage for fixed-fixed beams with a thickness of 2 *μ*m.

**Figure 14:** Pull-in voltage versus size effect for fixed-fixed beam with gap of 2.5 *μ*m, a thickness of 1 *μ*m, length of 300 *μ*m, and width of 0.5 *μ*m, for nonlinear geometry model.

**Figure 15:** Pull-in voltage versus size effect for cantilever beam with gap of 2.5 *μ*m, a thickness of 1 *μ*m, length of 300 *μ*m, and width of 0.5 *μ*m, for linear and nonlinear geometry model.

**Figure 16:** General ANN topology.

**Figure 17:** Comparing the theoretical and RBF neural networks pull-in voltages for silicon 110.

**Figure 18:** Comparing pull-in voltage of the microcantilever versus parameter *h*/*l* and *b*/*g* = 50 with RBF models.

**Table 1:** Geometrical parameters and material properties of microbeam.

Material properties		Geometrical dimensions			
*E* (GPa)	*v*	*L* (*μ*m)	*B* (*μ*m)	*h* (*μ*m)	*g* (*μ*m)
77	0.33	100–500	0.5–50	0.5–4	0–30

**Table 2:** Beam geometry and pull-in voltage for verification analysis.

Test number	*L* (*μ*m)	*b* (*μ*m)	*h*/*l*	*g* (*μ*m)	*V*_PI_ (volt)
1	75	0.5	4	0.5	0.179
2	100	5	6	1	2.44
3	125	10	8	1.5	7.31
4	150	20	10	2	16.82
5	175	25	12	2.5	26.78
6	200	30	14	3	40.27
7	225	35	16	3.5	53.84
8	250	40	18	4	68.01
9	275	45	20	4.5	84.53
10	300	50	22	5	103.62

**Table 3:** The effects of different number of hidden neurons on the RBF network performance (*S* = 3).

Number of hidden neurons	Average error (%) in predicting *V*_PI_ with newrbe function	Average error (%) in predicting *V*_PI_ with newrb function
16	8.87	7.3
18	9.66	10.77
20	4.55	6.08
22	12.32	14.71
24	12.89	15.16
26	13.78	16.24

**Table 4:** Comparison of *V*_PI_ calculated and predicted by the RBF neural network model.

Test number	*V*_PI_ (volt)			*V*_PI_ (volt)		
	Calculated	RBF model (newrbe)	Error (%)	Calculated	RBF model (newrb)	Error (%)
1	0.179	0.19	8.49	0.179	0.18	3.78
2	2.44	2.47	1.34	2.44	2.70	10.97
3	7.31	7.68	5.12	7.31	7.81	6.93
4	16.82	16.88	0.38	16.82	17.27	2.71
5	26.78	27.47	2.59	26.78	27.76	3.69
6	40.27	41.96	4.20	40.27	43.20	7.29
7	53.84	54.80	1.79	53.84	54.96	2.09
8	68.01	70.64	3.88	68.01	75.06	10.38
9	84.53	85.43	1.07	84.53	88.40	4.59
10	103.62	120.89	16.67	103.62	113.75	9.78

## References

[1] Khatami I, Pashai MH, Tolou N (2008). Comparative vibration analysis of a parametrically nonlinear excited oscillator using HPM and numerical method. *Mathematical Problems in Engineering*.

[2] Gasparini AM, Saetta AV, Vitaliani RV (1995). On the stability and instability regions of non-conservative continuous system under partially follower forces. *Computer Methods in Applied Mechanics and Engineering*.

[3] Osterberg PM, Senturia SD (1997). M-test: a test chip for MEMS material property measurement using electrostatically actuated test structures. *Journal of Microelectromechanical Systems*.

[4] Osterberg PM, Gupta RK, Gilbert JR, Senturia SD Quantitative models for the measurement of residual stress, poisson ratio and young’s modulus using electrostatic pull-in of beams and diaphragms.

[5] Sadeghian H, Rezazadeh G, Osterberg PM (2007). Application of the generalized differential quadrature method to the study of pull-in phenomena of MEMS switches. *Journal of Microelectromechanical Systems*.

[6] Salekdeh YA, Koochi A, Beni YT, Abadyan M (2012). Modeling effect of three nano-scale physical phenomena on instability voltage of multi-layer MEMS/NEMS: material size dependency, van der waals force and non-classic support conditions. *Trends in Applied Sciences Research*.

[7] Batra RC, Porfiri M, Spinello D (2007). Review of modeling electrostatically actuated microelectromechanical systems. *Smart Materials and Structures*.

[8] Lin WH, Zhao YP (2008). Pull-in instability of micro-switch actuators: model review. *International Journal of Nonlinear Sciences and Numerical Simulation*.

[9] Koiter WT (1964). Couple-stresses in the theory of elasticity: I and II. *Proceedings of the Koninklijke Nederlandse Akademie van Wetenschappen B*.

[10] Mindlin RD, Tiersten HF (1962). Effects of couple-stresses in linear elasticity. *Archive for Rational Mechanics and Analysis*.

[11] Toupin RA (1962). Elastic materials with couple-stresses. *Archive for Rational Mechanics and Analysis*.

[12] Anthoine A (2000). Effect of couple-stresses on the elastic bending of beams. *International Journal of Solids and Structures*.

[13] Yang F, Chong ACM, Lam DCC, Tong P (2002). Couple stress based strain gradient theory for elasticity. *International Journal of Solids and Structures*.

[14] Xia W, Wang L, Yin L (2010). Nonlinear non-classical microscale beams: static bending, postbuckling and free vibration. *International Journal of Engineering Science*.

[15] Asghari M, Rahaeifard M, Kahrobaiyan MH, Ahmadian MT (2011). The modified couple stress functionally graded Timoshenko beam formulation. *Materials and Design*.

[16] Rong H, Huang QA, Nie M, Li W (2004). An analytical model for pull-in voltage of clamped-clamped multilayer beams. *Sensors and Actuators A*.

[17] Heidari M, Beni YT, Homaei H (2013). Estimation of static pull-in instability voltage of geometrically nonlinear Euler-Bernoulli microbeam based on modified couple stress theory by artificial neural network model. *Advances in Artificial Neural Systems*.

[18] Kong S, Zhou S, Nie Z, Wang K (2008). The size-dependent natural frequency of Bernoulli-Euler micro-beams. *International Journal of Engineering Science*.

[19] Ma HM, Gao XL, Reddy JN (2008). A microstructure-dependent Timoshenko beam model based on a modified couple stress theory. *Journal of the Mechanics and Physics of Solids*.

[20] Gupta RK (1997). *Electrostatic pull-in test structure design for in-situ mechanical property measurements of microelectromechanical systems [Ph.D. thesis]*.

[21] Zhao J, Zhou S, Wang B, Wang X (2012). Nonlinear microbeam model based on strain gradient theory. *Applied Mathematical Modelling*.

[22] Freeman JA, Skapura DM (1992). *Neural Networks: Algorithms, Applications, and Programming Techniques*.

[23] Gao D, Kinouchi Y, Ito K, Zhao X (2005). Neural networks for event extraction from time series: a back propagation algorithm approach. *Future Generation Computer Systems*.

[24] Demuth H, Beale M (2001). *Matlab Neural Networks Toolbox, User’s Guide*.

[25] Shao H, Zheng G (2011). Convergence analysis of a back-propagation algorithm with adaptive momentum. *Neurocomputing*.

[26] Wasserman PD (1989). *Neural Computing: Theory and Practice*.

[27] Gholizadeh S, Samavati OA (2011). Structural optimization by wavelet transforms and neural networks. *Applied Mathematical Modelling*.

[28] Gholizadeh S, Salajegheh E (2010). Optimal design of structures for earthquake loading by self organizing radial basis function neural networks. *Advances in Structural Engineering*.

